This article has been retracted.

# A fuzzy model for content-centric routing in Zigbee-based wireless sensor networks (WSNs)

**DOI:** 10.1371/journal.pone.0286913

**Published:** 2023-06-15

**Authors:** Zhou He, Lian Chen, Feng Li, Ge Jin

**Affiliations:** 1 State Key Laboratory of Particle Detection and Electronics, University of Science and Technology of China, Hefei, China; 2 Department of Modern Physics, University of Science and Technology of China, Hefei, China; TU Wien: Technische Universitat Wien, AUSTRIA

## Abstract

WSN is one of the most efficient technologies in intelligent communication and because of its advantages, this technology has been utilized in various applications. By using WSNs, different types of data can be collected and analyzed in wide environments. The high variety of applications and types of data available in this network can cause several challenges about heterogeneous data routing. This research, presents a Fuzzy Model for Content-Centric Routing (FMCCR) in WSN to solve these challenges. The performance of FMCCR is based on two basic steps: "topology control", and "data transmission through content-centric and fuzzy logic-based routing algorithm". In the first step of FMCCR, the network topology is constructed. In the second step of the proposed method, data transmission paths are determined based on network topology and content type, and data transmission is performed. The performance of FMCCR has been evaluated in a simulation environment and the results have been compared with previous algorithms. The results show that FMCCR reduce energy consumption and improve the traffic load distribution in the network in addition to increasing the network lifetime. According to the results, FMCCR can increase network lifetime at least 10.74% and at the same time, deliver at least 88.1% more packets through the network, compared to previous methods. These results, prove the efficiency of the proposed method for using in real-world scenarios.

## 1. Introduction

WSN is one of the most key existing technologies based on wireless communication. Advantages of WSN such as scalability, high flexibility, the ability to be used in various environments, etc. have led to the increasing use of these networks in various fields. This technology can provide the possibility of monitoring wide environments without the presence of human agents. The basis of this technology is based on wireless radio waves that allow different devices to communicate with each other through these waves [1]. With the introduction of new architectures such as the Internet of Things (IoT), WSN applications entered a new phase and caused new issues such as supporting a large number of sensor nodes and a high variety of data types in the network [2]. However, transmission and management of a wide range of heterogeneous data in WSNs based on the IoT is a challenge that has caused the inefficiency of previous routing algorithms in this network [3]. WSNs can be used for many applications in various industrial fields, including environmental monitoring, urban services, surveillance and security applications, etc. However, collecting large amounts of data from such networks, including figures, images, video, etc., often causes traffic congestion in some areas [4]. CCR is one of the solutions introduced to solve this problem and achieve routing goals in WSNs based on the IoT.

In CCR, the appropriate path for data transmission is determined according to its content. In this method, related data are processed by intermediate nodes, and aggregation is done based on the content of related data. Hence, network traffic is effectively reduced. As a result, a significant reduction in delay can be achieved. In addition, redundant data transmission after data collection can be ignored, which mainly reduces the energy consumption on wireless communication and thus saves battery life [5]. This method, despite improving the network performance in general, does not have enough efficiency in situations where the variety of data is high. Because in previous CCR methods, the decision to aggregate data must be made specifically for each type of content. In real applications of IoT, a thing can transmit any type of content (temperature, humidity, sound, vibration, etc.). This high diversity can make the act of combining data in previous strategies difficult [6].

To solve this limitation, fuzzy logic is used in this article to decide how to aggregate data. The main contributions of the current article is twofold:

- This paper presents a new fuzzy model to make decisions about data routing based on the type of content being transmitted. The proposed fuzzy inference system eliminates the dependence of the CCR algorithm performance on the types of data content and increases network flexibility.
- This paper proposes a new routing mechanism for WSNs which causes data transmission routes to be determined according to the type of content, which is effective in reducing data redundancy and increasing network life.

The diagram of research workflow is illustrated in Fig 1. As shown in this diagram, this research started with identifying problem. Based on the identified research problem, the research objectives were implemented. These objectives include: improving the mechanism of CCR in WSNs independent from variety of data types, maximizing WSN lifetime, and uniform traffic distribution over network. According to the research objectives, the proposed method was designed and then, its efficiency was evaluated in a simulated environment. The parameters of the model were modified, until the research goals were met. Finally, the simulation results were analyzed and discussed.

**Fig 1:** The diagram of research workflow.

The rest of the article is organized as follows: In section 2, some previous related studies are reviewed. In section 3, the details of the FMCCR are presented, and in section 4, the results of the FMCCR implementation are discussed. Finally, in section 5, the research findings are summarized.

## 2. Literature review

Routing in WSNs is one of the most popular research topics in the field of wireless networks. So far, various methods for routing in WSNs have been presented, and in this section, a brief review of some of these research works are discussed. In [7], a fault-tolerant routing algorithm for WSNs was presented, using Genetical Swarm Optimization (GSO) algorithm, which is a combination of Genetic Algorithm (GA) and Particle Swarm Optimization (PSO). In this method, the energy, coverage, communication cost, and proximity criteria are used to select the cluster head nodes. Also, the GSO algorithm is used to determine data transmission routes.

In [8], a clustering and routing algorithm based on the combination of PSO and Gravitational Search Algorithm (GSA) was introduced. This method has improved the convergence of the PSO algorithm by combining it with the GSA algorithm. Comparing the results of this combination with the simple PSO algorithm shows the improvement of its convergence speed; however, this method also uses a centralized solution in the base station to determine the optimal routes.

Layered Energy Balanced Unequal Clustering and Routing (LEBUCR) method in [9] adopts an Unequal clustering mechanism combined with intra-cluster multi-hop routing. Through a time-based competitive clustering method, LEBUCR segments all nodes into asymmetric clusters where cluster heads can allocate more energy for intra-cluster communication to avoid the problem of congestion points.

In [10], a clustering and routing method in WSN called ICSHS was proposed, using the combination of cuckoo and harmony search algorithms. In this method, the network clustering structure is generally constructed using the cuckoo search algorithm. In this way, the different network nodes clustering types are checked and the degree of fitness in the current clustering is calculated for each case.

In [11], differential clustering was used for routing in WSNs. Differential clustering algorithm solves the problem of stray nodes in the network, and in addition, it can be effective in the balanced distribution of energy consumption over the network. In [12], the problem of cluster head selection and routing in WSN is considered as an optimization problem, and a new optimization algorithm called Cuckoo Insisted-Rider Optimization Algorithm (CI-ROA) was used to solve it. This optimization algorithm is a combination of Cuckoo Search (CS) and Rider Optimization Algorithm (ROA). In this method, criteria such as energy, distance, and delay are considered as the goals of the optimization algorithm.

In [13], an approach similar to the method presented in [7] was used for clustering and routing in a WSN. The authors named their method GA and PSO based hybrid (GAPSO-H), which is a combination of GA and PSO. In this method, GA is used to select the cluster head nodes and PSO is responsible for determining the data transmission paths.

In [14], a fuzzy inference system was used for secure routing in WSNs. This method uses a rule-based fuzzy model for clustering and routing in the sensor network. Along with this routing algorithm, a fuzzy algorithm based on time and distance was used to monitor the activity of each cluster member and determine the attacking nodes in the sensor network.

In [15], a routing algorithm with congestion control capability in WSNs was introduced. In this method, sensor nodes are first clustered using a combination of K-means and greedy search algorithms. Then the Firefly Optimization (FFO) algorithm is used to control the data rate of the sensor nodes. Finally, the data transmission routes are determined through the Ant Colony Optimization (ACO). In [16], a trust-based routing algorithm in WSNs was proposed. In this algorithm, Chicken-Dragonfly (CHicDra), selects cluster head nodes and determines reliable routes based on criteria such as comprehensiveness, stability, successful forwarding rate, and accessibility.

In [17], an energy efficient routing algorithm, called Energy-aware Proportional Fairness Multi-user Routing (EPFMR), was presented for using in WSNs. This routing algorithm tries to determine the best data transmission routes based on communication records between sensor nodes, and for this, it uses a greedy method to measure the energy consumption in multi-hop routes.

In [18], the combination of GA and Equilibrium Optimizer (EO) algorithm was utilized for clustering and routing in WSN. The first algorithm selects cluster head nodes and the second algorithm determines data transmission routes in the network.

The method presented in [19] is a clustering and routing algorithm in WSNs using a combination of fuzzy logic and optimization algorithms. In this method, a fuzzy model is used to form an unequal clustering structure in a WSN. In the unequal clustering method, the radius of clusters are not equal and the congested areas of the network often contain clusters with a smaller radius so that the load balancing and energy consumption over the network can be improved. After the construction of the cluster structure, the Glow-worm Swarm Optimization (GSO) algorithm selects the data transmission routes. This algorithm tries to determine the routes based on the data context.

Research in [20], proposed an optimization-based clustering and routing algorithm for WSNs. In this method, nodes of WSN are clustered using Adaptive Sailfish Optimization (ASFO). The optimization goals in this clustering algorithm include: energy, distance and latency. This research also introduces an energy-efficient cross-layer-based expedient routing protocol (E-CERP) for determining the paths in WSN. In [21], a secure routing and clustering method for WSNs is introduced which focuses on selecting stable cluster heads and routing paths. This method, uses a combination of Quadrature LEACH (Q-LEACH) and Multi-Hop LEACH (MH-LEACH) for constructing the clustered structure of the WSN.

Research in [22], has focused on clustering and routing in WSNs with mobile sinks. This method, uses a score function for cluster head identification, and controls the movement of sink nodes using two parameters based on density and delay. In [23], Genetic Algorithm (GA) has been used for unequal clustering and routing in WSNs. In this method, first GA is used for selecting cluster heads based on: energy, distance and inter-cluster separation criteria. Then, a routing algorithm based on GA is introduced for multi-hop routing among cluster heads which selects routes using energy, distance and number of hops.

## 3. The proposed method (FMCCR)

The algorithm presented in this research provides a new structure for topology control and CCR in WSNs. In this research, a WSN environment is considered based on Zigbee with a limited movement range of nodes and each node has a unique and unchanging ID. The set of network nodes is shown as *M* = {*M*_1_, *M*_2_,…,*M*_*N*_} where N is the number of network nodes. Each node has a fixed data type with a specific volume and its content changes in different time intervals. The network data set is defined as *D* = {*D*_1_, *D*_2_,…,*D*_*N*_}. It is assumed that each node has limited memory and according to its memory capacity, it can store data from set D in its memory. The network nodes have different characteristics and as a result, the network structure is heterogeneous. Neighboring two nodes means that they are covered by radio communication range of each other, and two wireless nodes that are not in the same neighborhood are called disconnected. The following definitions are used in describing the concepts of the proposed method:

Definition 1: For graph G = (V,E) where V is the set of vertices and E is the set of edges, a Dominating Set (DS) is a subset of the vertices of the graph *S*∈*V* in which each vertex of graph G is either a member of S or connected to it.

Definition 2: A Connected Dominating Set (CDS) is a state of DS in which all vertices are connected.

The model used to calculate the amount of energy consumed in communication between nodes is based on the model presented in [24]. In this model, the amount of energy used to transmit N bits of data between two nodes is obtained as follows [24]:

$$E_{TX}\left(N,d\right)=N\times (E_{elec}+E_{amp}.d^{n})$$ (1)

Where:

$$n=\left\{\begin{array}{cc} 2, & if\;d\leq d_{0}\\ 4, & if\;d>d_{0} \end{array}\right.$$ (2)

And:

$$d_{0}=\sqrt{\frac{E_{fs}}{E_{amp}}}$$ (3)

In (1), d is the distance between two nodes, *E*_*elec*_ is the energy consumed per bit in the transmitter and receiver circuits, and *E*_*amp*_ is the transmitter amplifier parameter for multipath fading. In (3), *E*_*fs*_ denotes the transmitter amplifier parameter for free space. Also, the energy consumption to receive N bits of data is calculated according to (4):

$$E_{RX}\left(N,d\right)=N\times E_{elec}$$ (4)

Before addressing the process of CCR in FMCCR, it is necessary to state the assumptions used in its design. The assumptions used in the rest of this section are:

- The location of nodes in the network is random and uniform, and some network nodes are mobile. Also, the position of the base station in the network is assumed to be fixed.
- The strength of the received signal in wireless communication has a direct relationship with the distance between the transmitter and the receiver. Therefore, the distances between the nodes can be estimated through analyzing the received signal strength.
- The assumed network uses Zigbee standard characteristics to control the performance of the sensor nodes. Thus, the data rate of each sensor node is determined based on the allowed values in this standard.
- Each active sensor node in the network can analyze the contents of the packets in its buffer memory. In this way, a node can recognize the type of content being routed and report to other nodes.

Based on the described network model and assumptions, the details of FMCCR are explained as follows. The performance of FMCCR is based on two main phases:

1. Topology control
2. CCR based on fuzzy logic

In the following, each of these steps is explained.

### 3.1. Topology control

The first step in the FMCCR is to construct and control the network topology. The proposed topology control algorithm performs the topology construction using the CDS solution. Fig 2 shows the DS and CDS for a hypothetical graph.

**Fig 2:** (a) DS, (b) CDS for a hypothetical graph.

As shown in Fig 2, for the assumed graph, the set DS = {c, e} can be considered as a DS in which each vertex is connected to one of the members of this set. The formed DS is not connected and therefore cannot be used as the communication structure in a wireless network.

By adding node *d* to the DS, it can be turned into a CDS, which is suitable for use as a network communication topology. It should be noted that several CDSs can be created for the assumed graph, but in the applications of wireless communication, the construction of the minimum CDS is desirable. The purpose of the topology construction step in FMCCR is to determine an optimal CDS as a communication infrastructure between network sensor nodes. In [25], a distributed algorithm was presented to find the CDS in a connected graph. The algorithm presented in this section is designed based on the proposed scheme in [25].

The first step of the topology construction process is to identify the neighbors for each node. For this purpose, each node with sufficient energy informs its neighbors about its presence by broadcasting a Hello message. Any neighboring node that receives this message adds the transmitter node to its neighbor set.

By doing this process of all the active nodes of the network, each wireless node can identify the set of active nodes located in its neighborhood. After this process, the topology construction algorithm starts by marking all the active nodes with zero. In the following, the base station as the starting node of the topology construction process is marked with number 2, and all its neighbors are marked with number 1.

Then, in the next step of the topology construction process, a node marked with number 1 is selected, which has the largest number of neighbors marked with zero, and then the selected node is marked with number 2 and its neighbors are marked with the number 1. This process will be repeated until all the active nodes are marked with number 1 or 2. In this way, the CDS includes the nodes marked with number 1. So, the topology construction algorithm used in FMCCR could be implemented in the following steps:

1. Every active node that has at least one neighbor is marked with zero.
2. The base station is considered as the starting point of the topology.
3. The starting node of the topology is marked with number 2 and its neighbors with number 1.
4. Until all the active nodes are marked with one of the numbers 1 or 2, the following step is repeated:
  - Node with sign 1 that has the largest number of neighbors with sign 0; is selected
  - The selected node is marked with number 2 and its neighbors with number 1
5. The set of all nodes marked with the number 2, forms the CDS.

After performing the above steps, network topology connections will be formed. This topology specifies the communication paths between the active sensor nodes and the base station. Since the formed topology is a CDS; therefore, there may be more than one route between each node and the base station. It should be noted that the formed topology structure is stable only for the minimum lifetime of network connections, and if the first connection is interrupted, access to a part of the network may not be possible. For this reason, after a period equal to the minimum expected lifetime in network connections, the topology construction process is repeated:

$$T_{i,j}=\frac{d.\text{cos}(\varphi_{ij})+\;\sqrt{r^{2}-d^{2}\;{\text{sin}}^{2}\left(\varphi_{ij}\right)}]}{v_{ij}}$$ (5)

$$v_{ij}=\sqrt{{\left(v_{i}\;\text{cos}\left(\varphi_{i}\right)-v_{j}\;\text{cos}\left(\varphi_{j}\right)\right)}^{2}+{\left(v_{i}\;\text{sin}\left(\varphi_{i}\right)-v_{j}\;\text{sin}\left(\varphi_{j}\right)\right)}^{2}}$$

$$\varphi_{ij}={\text{tan}}^{-1}\frac{v_{i}\;\text{sin}\left(\varphi_{i}\right)-v_{j}\;\text{sin}\left(\varphi_{j}\right)}{v_{i}\;\text{cos}\left(\varphi_{i}\right)-v_{j}\;\text{cos}\left(\varphi_{j}\right)}$$

In (5), *T*_*i*,*j*_ specifies the expected lifetime for the communication link of two neighboring nodes *i* and *j*, *v*_*i*_ indicates the movement speed of node *i*, and *φ*_*i*_ specifies the movement angle of this node. Also, *r* represents the radio communication range of the node and *d* represents the distance between two nodes *i* and *j*, which is estimated by sampling the received signal strength. After constructing the network topology, route selection and data routing operations are performed. Choosing the right route based on the content is done in the second step of the proposed method using a solution based on the content-centric routing algorithm and fuzzy logic. In the following, this step of FMCCR is explained.

### 3.2. CCR based on fuzzy logic

CCR is a distributed process. When the node enters the network, based on the topology, it discovers different routes to reach the destination based on the construction process described in the previous step. Then, each active node in the network, in case of sensing an event and creating data, sends a local query message to the neighboring nodes (child nodes in the topology structure) and chooses the appropriate step to forward the data based on its content type. This query message includes the type of data content. After sending the query message, the eligible candidate nodes respond to the transmitter node with an ACK message, which contains the information required by the object function, such as the responding ID and the estimated lifetime of the responder node (if data is sent to it). By using this information as the input of the objective function, the rankings of the candidate nodes are performed, and one of the candidates having the highest ranking is selected as the destination node in this step, and finally, the target node updates the routing table and this procedure continues until the data reaches the base station. As a result of this process, a tree topology for multiple traffic content types can be dynamically updated. The operation of CCR in FMCCR includes two main functions:

1. Activation function
2. Objective function based on fuzzy logic

The activation function makes decisions for the objective function in CCR. The nodes’ queries cause the neighbors to provide some of their information (such as data traffic status, remaining battery power level, and content in their routing tables). With this information as the input of the objective function, the ranking of the candidate nodes is done using a fuzzy inference system and the node with the highest ranking is selected for the corresponding content path. Each of these functions is described below.

#### 3.2.1. Activation function

In dynamic network environments, most routing protocols periodically update their routing information. This action imposes additional control costs in the routing process. In networks with limited resources and weak connections, these messages should be controlled to save the node’s battery power. In the proposed method, the probability of executing the objective function at time t is calculated with the probability of *P*_*t*_. This probability is calculated independently on each node and does not require local or global network information. The probability of *P*_*t*_ is obtained from (6):

$$p_{t_{i}=\text{min}\;\;\{(\sum_{t_{p}}^{t_{i}}\;|\;d_{k}|)\;\times \;P_{init\;},1\}}$$ (6)

In (4), d_k_ shows the change in the traffic content of each node over time. *t*_*i*_ and *t*_*p*_ represent the current time and the previous time respectively. *P*_*init*_ is the default value of the objective function execution probability and is constant. Therefore, the probability of executing the objective function increases if a large value for d_k_ is obtained according to the changes in the generated content. On the other hand, when the network is in a static state (d_k_ is small), the value of $P_{t_{i}}$ decreases. Finally, if there is no change in the type of node content, the value of $P_{t_{i}}$ becomes *P*_*init*_. This probability adjustment process effectively reduces overhead and ensures that routing tables are updated even in a static environment.

#### 3.2.2. Objective function based on fuzzy logic

The objective function F is executed on a target node such as i, to find the most suitable node j (next step) for each data content such as K among the (N) neighboring candidates. Since in CCR, data traffic is separated by its content type, the target node considers a separate routing input for each unique content and updates it using the objective function. In FMCCR, a fuzzy inference system is used as the objective function. The structure of this fuzzy model is shown in Fig 3.

**Fig 3:** The proposed fuzzy model for objective function in CCR.

According to Fig 3, the fuzzy model used as the objective function is a Mamdani fuzzy inference system with two input variables, one output variable, and 9 fuzzy rules. The membership functions of input and output variables in the proposed Fuzzy Inference System (FIS) are illustrated in Fig 4.

**Fig 4:** The membership functions of input and output variables in the proposed FIS.

In Fig 4, “Traffic Reduction” and “Stability” denote the first and second input variables of the proposed FIS; while, “Priority” is its output variable. The first input of this fuzzy system describes the amount of data traffic reduction through the aggregation process and has three membership functions "low", "medium" and "high". In the proposed fuzzy model, the data traffic reduction input is described using the following relationship:

$$I_{1}=\frac{V_{p}-V_{a}}{V_{p}}$$ (7)

In the above relationship, *V*_*p*_ represents the volume of data traffic being exchanged before its allocation to the current node and *V*_*a*_ represents the volume of data traffic being exchanged after its allocation to the node and aggregation. the above relationship determines the amount of data traffic reduction with the forward delivery of current data to each of the candidate nodes.

The second input fuzzy variable in the proposed model is the communication quality which estimates the increase in the lifetime of the local network. This input variable also has three membership functions "low", "medium" and "high" and is described using the following relationship:

$$I_{2}=\frac{E_{p}-E_{n}}{E_{min}}$$ (8)

In (6), *E*_*p*_ represents the current energy of the candidate node and *E*_*n*_ specifies the estimated energy for this node after forwarding data, and *E*_*min*_ represents the lowest energy level available in the network. As a result, by using the second input variable in the fuzzy system, it is tried to select the candidate nodes with the lowest energy loss for data transmission and aggregation.

By using the described fuzzy variables, the output of the fuzzy system is determined as a fuzzy variable that indicates the priority of each candidate node for forwarding data. In the proposed method, nodes that have the highest priority determined by the fuzzy model are selected for routing and packet aggregation. The rules used in the proposed fuzzy inference system for prioritizing candidate nodes are given in Table 1. Based on these rules, the objective function based on fuzzy logic tries to select nodes for data aggregation and CCR that have the lowest traffic and energy consumption.

**Table 1:** Rules of the proposed fuzzy inference system for the objective function in CCR.

Rule ID	Input Variables		priority (Output)
	TrafficReduction	Stability	
**1**	low	Low	very low
**2**	low	medium	very low
**3**	low	High	low
**4**	medium	Low	low
**5**	medium	medium	medium
**6**	medium	High	high
**7**	high	Low	medium
**8**	high	medium	high
**9**	high	High	very high

## 4. Results

The simulation was done in MATLAB. The network simulation parameters are based on the Zigbee standard specification. The model used to calculate the amount of energy consumed in communication between nodes is based on the model presented in [24] and (1) and (2). In this energy model, the amount of energy consumed per bit in the transmitter and receiver circuits is $E_{elec}=50\frac{nJ}{bit}$ and the energy consumed per bit in the RF amplifier is ${\;E}_{amp}=0.0013\frac{pJ}{bit\times m^{2}}$. Also, the transmitter amplifier parameter for free space was chosen as $\;E_{fs}=100\frac{pJ}{bit\times m^{2}}$; and therefore *d*_0_ = 87.70 *m*. All the assumptions stated in the network model were used in the simulation environment. The most important parameters used in the simulation environment are shown in Table 2.

**Table 2:** Simulation parameters.

Value	Parameter
200x200	Dimensions of the environment
Random Uniform	Distribution of nodes in the environment
Center of area (100,100)	Base station location
100 heterogeneous wireless nodes	Number of nodes
0.5 J	The initial energy of each node
Random between 20 and 30 meters	Radio range for a communication step
3 types of content that cannot be aggregated and have volumes of 1.5, 2, and 2.5 kilobits for each data report packet	Number of content types

Based on Table 2, three different types of content with volumes of 1.5, 2, and 2.5 kilobits are considered and the aggregation rate of these contents is set to $\frac{1}{M}$. This means that by receiving M packets with the same content, a node produces an aggregation packet with the same volume as the primary packets by performing calculation operations such as averaging. Also, none of the existing types of content can be combined. Fig 5 shows an example of a content-centric topology for an assumed network with 100 nodes and three types of content.

**Fig 5:** An example of topology based on the content formed for the assumed network.

As shown in Fig 5, the topologies formed for different types of content in the proposed method are unique. This means that FMCCR forms the topology structure by using the content analysis solution of data flowing in the network, as well as considering the ability of data processing by intermediate nodes. This solution increases efficiency in structures with diverse contents. In the following, the impact of this structure on the performance of FMCCR is investigated.

In this experiment, the network lifetime of FMCCR is checked and the results are compared with GAPSO-H routing algorithms in [13] and EPFMR in [17]. To maintain fairness in making comparisons, the initial state of all sensor nodes and the formation pattern of environmental events are considered the same for all methods. Network lifetime is one of the main criteria for checking the efficiency of routing algorithms. In this experiment, random events occur at different points in the network. Active nodes close to this event receive its information and send it to the data collection center. It should be noted that each node can produce and aggregate a specific type of content, and for non-processable types of content, only the transmission is performed. By continuously repeating these actions, the energy of the network nodes gradually decreases, and after several rounds, the energy of the network nodes runs out. The goal of routing algorithms is to maximize the number of rounds in data transmission so that all active nodes in the network can be used the most. Fig 6 shows the number of alive nodes in the network for the number of rounds in FMCCR and the compared algorithms.

**Fig 6:** The number of alive nodes in the network for different number of rounds.

As shown in Fig 6, the lifetime of the network in FMCCR is longer than the compared methods. Based on the results obtained from this test, FMCCR has more alive nodes than the compared methods in its entire period of operation. The reason for this can be attributed to the use of topology based on the CDS in FMCCR. This solution makes the network nodes use a suitable structure to form a topology based on the final content. As a result, it can be said that FMCCR will have a longer lifetime by increasing the number of rounds. These results show the effectiveness of FMCCR in energy consumption and indicate that the use of the CDS structure in FMCCR can distribute the network load in a balanced way to prevent the premature exhaustion of a node’s energy. These conditions are shown in Fig 7. In this figure, the number of alive and inactive nodes in rounds 200, 400, and 1000 for FMCCR is displayed.

**Fig 7:** The number of alive and inactive nodes in rounds 200, 400, and 1000 for FMCCR.

The same results for the EPFMR method (as a method with closer performance to FMCCR) are shown in Fig 8.

**Fig 8:** The number of alive and inactive nodes in rounds 200, 400, and 1000 for the EPFMR method.

As shown in Figs 7 and 8, FMCCR works efficiently in more uniform distribution of energy consumption in addition to increasing the lifetime of nodes at different rounds. So that, in round1000, FMCCR was able to maintain the connection of a large number of nodes with the central node, but in a similar situation and in the compared method, parts of the network lost their connection with other nodes. and the network is segmented.

In the following, the amount of energy consumed by all nodes is evaluated in FMCCR, and the results are compared with other methods. Fig 9 shows the total energy consumed in each round by all the nodes.

**Fig 9:** Total energy consumed in each round by all nodes.

As the simulation results show in Fig 9, the amount of energy consumption in FMCCR is lower than the compared methods. This has made the network more efficient and increased its lifetime during the simulation. The lower energy consumption in the performance of FMCCR can be attributed to the use of the CDS topology structure in the first step of FMCCR. As shown in Fig 9, in round 1740, the total energy consumption of FMCCR increases at once.

The same operation is repeated in round 1260 for the EPFMR method. The reason for the sudden increase in energy consumption at these points is the disconnection of a part of the network from the central areas. These areas are visible in the figure. In this case, which is called network segmentation, the stray nodes have to communicate with distant neighbors and as a result, they consume much more energy to send data. Nevertheless, the uniform distribution of energy consumption in FMCCR has caused the network segmentation process to occur later than the compared method. Also, the residual energy of the network per round is shown in Fig 10.

**Fig 10:** The residual energy of the network per round.

As the results of Fig 10 show, the amount of residual energy in FMCCR is higher than the residual energy in the compared methods for all rounds. Therefore, it is clear that FMCCR works much more efficiently in energy consumption. In this figure, the points of occurrence of segmentation which causes the rapid energy loss of network nodes are marked.

In the following, the number of packets exchanged between different nodes of the network is examined. Fig 11 shows the number of successfully delivered packets in the network for different rounds in the simulation.

**Fig 11:** The number of successfully delivered packets in the network for different rounds.

As shown in Fig 11, FMCCR can transmit data packets about two times more than the EPFMR method to the base station. The reason for this is that by repeating the simulation rounds, the number of active nodes of FMCCR exceeds the compared methods, and as a result, the number of exchanged packets in FMCCR increases. Also, after round 1200, the number of active nodes in the central areas of the network is reduced in EPFMR method and the traffic load is imposed on a small number of remaining nodes. In this case, the probability of memory overflow and data loss increases. Whereas in FMCCR, there are still enough nodes for sending data and routing. This efficiency in delivery is the result of using the routing algorithm presented in FMCCR. In addition to reducing energy consumption during data routing, this algorithm can transmit the number of more data packets between the network nodes by properly distributing the load.

At the end of this section, the amount of activity of nodes to send data packets in the network is examined. An effective method for distributing the load over the network should prevent sending too much data to a node so that the energy level of that node does not drop at once. Fig 12 shows the load imposed on each node for forwarding data. The first and second dimensions shown in the diagram are the horizontal and vertical coordinates of the network environment and each column represents the amount of load imposed on the node according to its position in the network.

**Fig 12:** Load imposed on each node for forwarding data according to the position of that node in the environment.

Considering that the database station is located in the center of the environment, as shown in Fig 12, the proposed method avoids imposing a heavy load on a node near the base station, and data packets are sent through different nodes in the neighborhood of the base station. This solution ensures that the energy of a node does not decrease at once and increases the network lifetime.

In the continuation of this section, the effect of changes in the number of network nodes on the performance of the proposed method will be investigated. In these experiments, the efficiency of the proposed method has been compared with GAPSO-H [13] and EPFMR [17]. In this experiment, the number of network sensor nodes was changed in the range of 100 to 300 nodes and the criteria of network lifetime and the total number of delivered packets were evaluated. It should be noted that other simulation parameters are determined based on Table 2. In Fig 13, the lifetime of the network is illustrated versus changes in the number of sensor nodes. Also, Fig 14 depicts the number of delivered packets per these changes.

**Fig 13:** The network lifetime as a function of number of sensor nodes.

**Fig 14:** Delivered packets as a function of number of sensor nodes.

As shown in Fig 13, increasing the number of nodes will increase the network lifetime. Because, increasing the number of sensors means increasing the number of energy sources that can participate in the routing process and keep the network active for a longer time. But this lifetime increase will occur if the clustering and routing protocol is able to optimally use the energy resources of the sensors. These conditions for the proposed method can be clearly seen in Fig 13 and the proposed method prevents the loss of energy of the sensor nodes and further increases the network lifetime by efficiently clustering of WSN and routing between the cluster head nodes. Follows the network. By increasing the network lifetime, it is natural that more data packets can be successfully delivered in the network. This condition can be clearly seen in Fig 14. These results confirm that the proposed method works well both in efficient clustering of nodes and routing packets. Based on the results, the proposed method can increase the lifetime of the network by 10.74% compared to the EPFMR method and by 48.16% compared to the GAPSO-H method. On the other hand, the proposed method can increase the average number of delivered packets in the network by 88.1% compared to the EPFMR method and by 193.36% compared to the GAPSO-H method.

## 5. Conclusion

In this article, a CCR algorithm in Zigbee-based WSNs was presented. The proposed method performs the routing process during two phases of topology construction and path selection based on content analysis and fuzzy logic. In the proposed method, the network topology is formed based on the structure of the CDS. This structure guarantees the variety of routes between the sensor nodes and the base station, as well as routes durability, based on which the routing process can be carried out with a more balanced load distribution over the network. The proposed method also uses a fuzzy inference system to determine data transmission routes based on the content being transmitted through packets. This fuzzy system can construct unique paths for any type of data, so that the intermediate nodes in each route can participate in forwarding packets, in a more efficient manner. This process can significantly reduce the amount of data being transmitted over the network, which will result in a reduction in energy consumption and an increase in the network lifetime. The efficiency of the proposed method was evaluated in a simulated environment, in terms of energy consumption, number of delivered packets and load distribution. Also, the proposed method was compared with previous efforts. According to the results, the proposed method can increase network lifetime and number of delivered packets at least 10.74% and 88.1%, respectively.

In future works, by considering more criteria (input variables) in the proposed fuzzy inference system, its flexibility in the network can be improved. Also, the researchers will try to develop the proposed method and investigate its application in the IoT architecture. Thus, in future works the proposed method will be implemented in WSN-IoT networks.

## Supporting information

S1 Data (XLSX)
